The article "The Impact of Environmental Technology and Environmental Policy Strictness on China's Green Growth and Analysis of Development Methods" was published in 2022. Journal: J Environ Public Health.

# The Impact of Environmental Technology and Environmental Policy Strictness on China's Green Growth and Analysis of Development Methods

**DOI:** 10.1155/2022/1052824

**Published:** 2022-09-22

**Authors:** Yiming Wu, Yichao Zhang

**Affiliations:** Zhejiang A&F University, Hangzhou, Zhejiang 311300, China

## Abstract

Environmental technology and the stringency of environmental policies have a certain effect on green growth in the country, and the sustainable development of the environment under the influence of green growth requires the effective application of the environmental technology based on such institutional policies related to the environment. In this paper, the mutual effect of green growth on the ecological environment is fully analyzed to identify an intrinsic link between them. Based on the intrinsic link, policies related to environment protection and environmental technology are conducive to facilitating green growth while at the same time playing a continuous role in the improvement of the environment. Driven by the factors of scientific and technological innovation, it can boost the harmonious development of the economy and the environment. The empirical evidence has demonstrated that the appropriate environmental policy and environmental technology model can be identified with full understanding of the environmental policy and environmental technology. At the same time, the industry drive and technological innovation can also be taken as a strong support for the environmental policy and the environmental technology in accordance with the market demand through research from the perspective of the government, the market, and the general public. The stringency of environmental policies has substantially increased the requirements of environmental technology, and the innovation of environmental technology, the structure of economic organizations, and the level of development have a great effect on the green growth in the country.

## 1. Introduction

In the continuous progress of industrialization and urbanization, economic development has had a certain influence on the natural environment, and the issue of “pollution first and treatment later” is observed in the development process of developed countries. In comparison, the economic development level in the country is not high. However, the environmental problems have also gradually affected the routine activities of people and their quality of life. The pursuit of economic growth can lead to a serious decline in the efficiency of economic development and severe problems of environmental pollution. The capacity to ensure economic growth and environmental improvement has become a consensus of research scholars in many countries to achieve sustainable development and scientific development [1, 2]. With the improvement of environmental technology as a goal of economic growth, it is necessary to ensure the continuous improvement of environmental sustainability so that the economic development can have lasting momentum and a solid foundation for the steady development of society. However, as environmental protection in general lags behind economic construction, green growth activities are carried out in the context of the economic conditions and the living environment, which can be controlled in the form of monetary policies in the general direction, and at the same time, it can also be controlled in the form of setting restrictions in exploiting the living environment, promoting the implementation of green growth, and facilitating the efficient use of resources [3, 4]. The so-called green growth is a new form of green growth activity where computer Internet factors and digital technologies are combined with the traditional economy to achieve investment financing, payment and security business. However, in contrast to the traditional economy, the business of green growth is more convenient, universal, and highly efficient, which has the features of green growth itself, thus making it easy to achieve the purpose of joint development in the economy and environment. As a basic requirement and effective approach to modernize the national management system, the report of the 18th Party Congress pointed out that the environmental policy and environmental technology should be applied. Under the influence of environmental policy and environmental technology, the thinking of environmental policy will become the mainstream ideology of society in the future, and the environmental policy model will gradually become the basic approach adopted in national institution management, government management, and social management [5, 6]. At different historical moments in history, there are different priorities for the formulation of policies related to the environment. As a result, the content of legal thinking and the policy approach related to the environment can also present different features. In the present, the main focus of environment-related policy thinking is about adhering to the premise of legality in combination with the rule ideology, focusing on making judgment in under the premise of legality with the awareness of environment-related policy and paying attention to the procedural justice. Based on the so-called “environment-related policy thinking”, the power holder audits the environment-related policy concepts, carries out analysis, summarizes findings, makes judgment, and conducts reasoning in multiple dimensions such as detailed analysis, change, and coordination of problems that arise in the process of laws and regulations, legal principles, legal spirit, and legal thinking [7–9]. With the full awareness of the process of cognitive activity of decision-making thinking, it is necessary to use the environment-related policy thinking as the basis of the relevant environment awareness to achieve the harmonious development of the related theory for improve the environmental policies. It has played a guiding role in the improvement and practice of the regulatory system. The related environmental regulations, policies, and environmental technology are developed mainly based on the behavior patterns that emerge from the thinking of environment-related policies, and the communication channels of environment-related policies and environmental technology are the thorough manifestation of their contents and forms. At present, the environmental technology requires the enterprises engaging in the environmental technology to have the capacity to provide one-stop services, offers strong support in lives, and ensures that the greatest economic benefit can be obtained through the environmental technology, which is the overall goal in the work of environmental technology enterprises. For the regions with frequent records of green growth business in the previous period, it has indicated that the local level of communication technology and communication business capacity are relatively good. As the green growth is developed based on the Internet technology, the analysis on the green growth development evolution based on the environmental technology has an important effect. A sound green growth development evolution analysis system can accelerate the flow of environmental technologies, reduce costs, ensure the proper operation of services, while at the same time ensuring the implementation of effective management and use of resources [10, 11]. For the purpose of effectively improving the accuracy of the analysis of the evolution of the green growth development of the environmental technology process, an evaluation algorithm is used to analyze the evolution of the objectives for the green growth development in real time. At the same time, it will also bring more long-term benefits to each region of the country. He Bin developed a set of restriction threshold model, this model for each region of China to reflect on the role of green growth per capita and the effect of the state-owned economy on the improvement of the ecological environment. With regard to the proposed sustainable growth of economic development, the key is to make breakthroughs in the economic structure through the energy perspective of the analysis, which, in fact, is the current general environment and the existing situation. It has been verified that the green growth situation in the country is inseparable from the two main causes of pollutant generation and environment in each region of the country, especially for the domestic situation.

With the formulation of environmental technology and environmental policy in the country, scientific and reasonable evaluation is carried out on the practical effect of environmental policies and subsidies on making effective improvement, which can provide a certain reference and play a guiding role in the implementation of the relevant environmental policies. The application of environmental technology and environmental policy system can play a certain positive role in driving the rapid economic growth, the effective improvement of environmental quality, and the optimization of the environmental system.

## 2. Mechanism of the Dual Effects of Environmental Technology and Stringency of Environmental Policy

The environmental technology and the stringency of environmental policies can often be deemed as potential constraints that have a direct effect on the transaction expenses, costs, profits, and management effectiveness in the growth of a green economy [12, 13]. While changing the green growth in the country, with regard to safeguarding the rights and obligations of the economy as a whole, it can urge people to save energy and contribute to the stable economic growth and improvement of social welfare standards effectively. In general situations, the use of environmental technologies and the stringency of environmental policies has many advantages in driving the economic growth and facilitate the environmental improvement processes. In addition, the environmental technology and the stringency of environmental policies can change the internal management efficiency and macroeconomic configuration via a number of pathways, as shown in Figure 1.

For developing countries, green economy is not a new term. In the research process of green growth both at home and abroad, no uniform template has been formed yet; and the construction of a green growth model is not a quick fix, which needs to be continuously adjusted and improved in the process of practice. In the early stage of rapid economic development, it may have high economic costs and expenses, along with high social costs. Hence, green growth is a long process of gradual advancement. Combined with the analysis above, a green transformation strategy is established in this paper, as shown in Figure 2. Its framework is designed around the main objectives of development, the strategies to be adopted, the criteria for the tasks, and the guarantee measures. Through the application of the “double transformation, entrepreneurship, and innovation” approach, the fruits of economic growth can be shared to finally achieve the purpose of national wealth and welfare for all the people [13, 14].

The goal of green economic growth is to implement economic “transformation” and “innovation”. With economic “transformation” as a strategic plan, it focuses on two key influences: the paradigm shift in the economic development and the policy changes in government agencies. First, the ultimate goal and positioning of the government and enterprises in the growth of green economy are determined. The “innovation” is taken as the criterion of development strategy, and then, it is necessary to focus on two aspects, that is, the economic growth mechanism innovation and the science and technology innovation. The continuous progress in science and technology will provide a solid foundation for green growth, while the innovation and change in the mechanism and system will provide effective guarantee for the growth of green economy. The relevant index data are collected from the process of ecological environmental protection, and the feedback is given accordingly. The data obtained are used to analyze the operating status of the ecological environment, diagnose the causes of faults, and also monitor the causes of faults. Green growth has facilitated the upgrading of industrial structure by optimizing the allocation of credit funds, boosting the technological innovation of enterprises, and enhancing the demand of residents for consumption. In turn, it can further affect the interaction effect of economic system and the environmental system. With the innovation of science and technology as a driving force of green growth, it can create a virtuous cycle between green growth and environmental technology. With the innovation of science and technology as the key to green growth, through in-depth theoretical research and analysis, it can be known that the investment in science and technology can facilitate green growth and create a scale effect, which will promote productivity and sustainable development of the economy. With the driving force of green growth, technological innovation can be applied and transformed to achieve economic growth at a higher speed [15]. In the formulation of low-carbon emission reduction policies, it is necessary to address the issues in the basic resources, environmental pollution status, and industrial structure features in different regions, different areas, and the corresponding cities in detail, taking into consideration the basic situation of each country's own economic development and social situation effectively, the availability of energy and policies related to green growth in various countries to actively explore the allocation of pollutant emissions and renewable energy that are most suitable for the respective region and guide the whole society to save energy, improve energy efficiency, and alleviate the pollution to the environment. In the analysis process of the traditional economic and ecological environment, ecological protection and risk alert in real time is also a process of effective data collection and analysis of the ecological protection status.

## 3. Measurement and Evaluation of Green Growth in China

The accurate measure of economic growth is taken as an important research index for the empirical evidence of growth [16]. In this paper, with the EBM model as the basis, the directional distance function (DDF) is defined. In accordance with the definition, it can be derived that if there are m types of inputs (*i* = 1,…,*m*) and 3 types of outputs (*i* = 1,…, *s*) in *n* decision units (*j* = 1,…, *n*); then, the EBM model established can be expressed as follows:

(1) $$\begin{array}{c} \gamma^{*}=\min\mathrm{\theta -}\varepsilon_{x}\sum_{i=1}^{m}\frac{w_{i}s_{i}}{x_{i0}},\\ s.t.\theta x_{0}-X\lambda -s=0,\\ \lambda Y\geq y_{0},\lambda \geq 0,s\geq 0. \end{array}$$

Among them, *γ*^*∗*^ in the expression stands for the optimal efficiency value of the function, which should be comply with the condition of 0 ≤ *γ*^*∗*^ ≤ 1; *w*_*i*_ stands for the weight of the input economic factor *i*, which should comply with the condition of ∑_*i*=1_^*m*^*w*_*i*_=1(*w*_*i*_ ≥ 0, ∀*i*); *θ* stands for the efficiency value of the radial direction; *s*_*i*_ stands for the corresponding function slack variable of the *i*-th input economic factor; *ε*_*x*_ stands for the combined radial *θ* and the nonradial slack variables as function parameters; *λ* stands for the level of significance in the objective decision unit adopted. *X*={*x*_*ij*_} ∈ *R*^*m*×*n*^ stands for the input vector of the economy, and *Y*={*y*_*ij*_} ∈ *R*^*s*×*n*^ stands for the output vector of the function, which should comply with the condition of *X* > 0 and *Y* > 0.

The GML index can be expressed by the available production set across the world, which can effectively address the issues of nontransmissibility and linearity that are observed in the ML index [17, 18]. In this paper, the EBM model and the GML index are used to provide a forecast of the green growth. For the global producible set in the *t* period and the *t* + 1 period, the GML index can be expressed as the following equation:

(2) $$\begin{array}{c} {\text{GML}}^{t,t+1}\left(x^{t},y^{t},b^{t},x^{t+1},y^{t+1},b^{t+1}\right)=\frac{1+D^{G}\left(x^{t},y^{t},b^{t}\right)}{1+D^{G}\left(x^{t+1},y^{t+1},b^{t+1}\right)}. \end{array}$$

In equation (2), *b*^*t*^ and *b*^*t*+1^ represent the undesired output and the directional distance function *D*^*G*^(*x*^*t*^, *y*^*t*^, *b*^*t*^)=max{*β* : (*y*+*βy*, *b* − *βb*) ∈ *P*^*G*^(*X*)} of the decision unit *t* period and *t* + 1 period, respectively.

It is assumed that *S*_*t*_ and *S*_*t*+*n*_ stand for the green growth in the *t* frame and the *t* + *n* frame and the mathematical model can be established in accordance with the workflow as follows:

(3) $$\begin{array}{c} S_{t}=B_{t}\left(x,y\right)+V\left(x,y\right)+N_{t}\left(x,y\right),\\ S_{t+n}=B_{t+n}\left(x,y\right)+V\left(x+\Delta x,y+\Delta y\right)+N_{t+n}\left(x,y\right). \end{array}$$

In equation (3), *B*_*t*_(*x*, *y*) and *B*_*t*+*n*_(*x*, *y*) stand for the factors of green growth in the *t* frame and the *t* + *n* frame; *V* (*x*, *y*) and *V*(*x*+Δ*x*, *y*+Δ*y*) stand for the environmental technology in the *t* frame and the *t* + 1 frame; *N*_*t*_(*x*, *y*) and *N*_*t*+*n*_(*x*, *y*) stand for the external disturbances of green growth in the *t* frame and the *t* + *n* frame.

The difference value (Δ*S*_(*t*+*n*)/*t*_) for the *t* frame and the *t* + *n* frame can be obtained by using the real-time update algorithm for economic data, as shown in the following equation:

(4) $$\begin{array}{c} \Delta S_{\frac{\left(t+n\right)}{t}}=S_{t+n}-S_{t}=\left[B_{t+n}\left(x,y\right)-B_{t}\left(x,y\right)\right]\\ +\left[V\left(x+\Delta x,y+\Delta y\right)-V\left(x,y\right)\right]+\left[N_{t+n}\left(x,y\right)-N_{t}\left(x,y\right)\right]. \end{array}$$

In equation (4), [*B*_*t*+*n*_(*x*, *y*) − *B*_*t*_(*x*, *y*)]+[*V*(*x*+Δ*x*, *y*+Δ*y*) − *V*(*x*, *y*)] stands for the factor of green growth and [*N*_*t*+*n*_(*x*, *y*) − *N*_*t*_(*x*, *y*)] stands for the factor of external interference.

*K*(*x*, *y*) stands for the binary differential green growth based on the real-time update algorithm for economic data, as shown in the following equation.

(5) $$\begin{array}{c} K\left(x,y\right)=\left\{\begin{array}{c} 1,\Delta S\geq T\\ 0,\Delta S<T \end{array}\right. \end{array}$$

In equation (5), *T* stands for the threshold value.

If the green economy in the country is regarded as 1 in 2002, then the growth level of domestic green economy in 2003 is the product of the level of growth in 2002 and the GML index for the corresponding growth in 2003. In this way, the value for the provincial domestic green growth during the period from 2003 to 2014 can be calculated accordingly. The specific arithmetic results of the domestic green growth in the two regions on average, that is, domestic and the east, central, and west regions, are shown in Figure 3:

In accordance with the green growth curve in Figure 3, the mean value of green growth in the country gradually increased from 2003 to 0.951. However, in 2014, the value was merely 0.951. This suggests that the measured index has a great potential for improvement. According to the change in the curve, the economy has presented an upward trend in the periods from 2005 to 2008 and from 2010 to 2014, which is mainly manifested in the period of the “11th Five-Year Plan” and the “12th Five-Year Plan”. With limiting the emission of pollutants as a binding index, the national government has clarified the responsibility for environmental protection, which has improved the overall environmental effect in the region to a great extent. However, the green growth of various regions in China started to decline after the occurrence of the economic crisis in 2008. The mean values for the green growth in the country are 0.9115, 0.8603, and 0.8756 in the east, central, and west regions, successively. The mean values in the eastern provinces, regardless of Hainan, Liaoning, or Hebei Province, are all higher than the average level in the country. Hence, it can be determined that there is a relatively high level of coordination maintained between the economic growth and the environmental performance in the east region.

## 4. Analysis of the Results

Based on the dual impact mechanism of environmental technology and the stringency of environmental policies on green growth in China analyzed in the above section, the potential nonlinear relationship of the environmental technology and the stringency of environmental policies with green growth in China is taken into comprehensive consideration [19, 20]. In this paper, a quadratic term for the environmental technology and the stringency of environmental policies is introduced to establish an econometric model in the following to explore the direct effect of environmental technology and the stringency of environmental policies on green growth in China.

(6) $$\begin{array}{c} \ln\;{\text{GTFP}}_{it}=\beta_{1}\sum_{j=1}^{3}\ln\;{\text{ER}}_{jit}+\beta_{2}\sum_{j=1}^{3}\ln\;{\left({\text{ER}}_{jit}\right)}^{2}+\beta_{3}\ln\;{\text{TI}}_{it}\\ +\beta_{4}\ln\;{\text{FS}}_{it}+\beta_{5}\ln\;{\text{IS}}_{it}+\beta_{6}\ln\;{\text{FDI}}_{it}+\mu_{i}+\varepsilon_{it}. \end{array}$$

In equation (6), *i* and *t* stand for provincial and annual GTFP for green growth in China, respectively; its specific value is obtained based on EBM-DDF; the command and control type (cer), the market incentive type ER_*j*_ (mer) free contractual environmental technology and the stringency of environmental policies (ver). It can be observed from Figure 1 that the direct factors influencing green growth in China include technological innovation (TI), factor structure (FS), industrial structure (IS), and foreign direct investment (FDI). The definition and descriptive statistics of each variable are shown in Table 1.

In addition, for the purpose of further exploring the indirect effect of the stringency of environmental technologies and environmental policies on the green growth in China, the following econometric model is established by adding the interaction terms for the stringency of three environmental technologies and environmental policies with the technological innovation, factor structure, industrial structure, and FDI [21, 22].

(7) $$\begin{array}{c} \ln\;{\text{GTFP}}_{it}=\beta_{1}\sum_{j=1}^{3}\ln\;{\text{ER}}_{jit}*\;\ln\;{\text{TI}}_{it}+\beta_{2}\sum_{j=1}^{3}{\mathrm{lnER}}_{jit}*\;\ln\;{\text{FS}}_{it}\\ +\beta_{3}\sum_{j=1}^{3}\ln\;{\text{ER}}_{jit}*\;\ln\;{\text{IS}}_{it}+\beta_{4}\sum_{j=1}^{3}\ln\;{\text{ER}}_{jit}*\;\ln\;{\text{FDI}}_{it}+\mu_{i}+\varepsilon_{it}. \end{array}$$

In equation (7), ln  ER_*j*_*∗*  lnTI stands for the interaction term of the three environmental technologies and the stringency of environmental policies with the technological innovation; ln  ER_*j*_*∗*  lnFS stands for the interaction term of the three environmental technologies and the stringency of environmental policies with the factor structure; ln  ER_*j*_*∗*  lnIS stands for the interaction term of the two environmental technologies and the stringency of environmental policies with the industrial structure; ln  ER_*j*_*∗*  lnFDI stands for the interaction term of the two environmental technologies and the stringency of environmental policies with FDI.  Table 2 shows the direct effects of the two environmental technologies and the stringency of environmental policies on green growth in China. The economic analysis model established for each region is analyzed in depth to evaluate the development factors of the relevant economy and the influencing factors in the development of each regional economy and the environmental technology. The results indicate that the accuracy in the sustainability of green growth can be improved rapidly, which can also enhance the efficient utilization of economic resources. In an environment of green growth, the rapid restructuring of the economy in each region can play a complementary role for environmental protection. In the process of analyzing the green growth development and evolution based on the traditional environmental technology [3, 4], it generally focuses on the green growth development evolution analysis based on the environmental technology. As the two-dimensional map can only describe a relatively high level of environmental plane information, but it cannot provide the relatively complete information on economic data [5, 6], the result can be inaccurate. Through the establishment of a model to evaluate the influencing factors on the development and environmental technologies in each regional economy, the accuracy in the sustainability of green growth thus obtained can be rapidly improved. In addition, it can also facilitate the effective implementation of green growth in each domestic region. By comparing the specific practices of other green growth development and analyzing their commonalities and features in depth, the suitable pathway for green growth in China development is explored to provide solutions and a theoretical basis for the green growth development in the country.

The industrial structure (IS) has not presented the expected positive effect on green growth in China. The possible reason is that in the special stage of China's economy at present, it has determined the dependence of economic growth on heavy industry. Hence, it is a slow process to improve green growth in China simply by adjusting the industrial structure. The foreign direct investment (FDI) has significantly improved the green growth in China with the technology spillover and demonstration effects [23, 24].

Table 3 shows the indirect effects of three environmental technologies and the stringency of environmental policies on green growth in China. The effect of the environmental technology is analyzed in detail to explore the problems and defects of the green growth development process so that targeted training programs and effective improvement plans can be developed in a later stage. Green growth development has gradually become an essential research direction for urban environmental technology. Through the in-depth analysis of the typical green growth development models both at home and abroad, the commonalities and features of their development processes are explored to summarize the regularity and innovation in the process of facilitating green growth development effectively. In this paper, the evaluation algorithm is used to obtain high-precision green growth development objective analysis results effectively, which can meet the requirement for real-time analysis of green growth development.

From the perspective of the factor structure pathway, the positive coefficient of the interaction term suggests that the environmental technologies and the stringency of environmental policies will in turn force the upgrading of factor structure so as to promote a higher level of green growth in China. In general, the coefficient of the indirect effect of factor structure is larger than that of the other two pathways. This suggests that China is gradually lowering its dependence on traditional energy sources to improve the factor structure, which can be attributed to the progress made in the energy price reform at present, and a substitution relationship can be observed between labor and energy [25, 26].

In this paper, the effect of an increase in the intensity of environmental restrictions on the economy, welfare, and environment is demonstrated, as shown in Figure 1. In this way, real-time, rationalization, and precise monitoring of ecological environment improvement can be implemented to provide a sound theoretical basis for analyzing the decisions made by the relevant environmental protection testing departments, which is of great significance for improving massive environmental technologies that have been emerging constantly. The environmental technologies are analyzed in detail to explore the problems and defects of the ecological improvement process so as to develop training programs and improvement plans subsequently. In the analysis on the improvement of the traditional ecological environment, the ecological environment improvement and real-time risk alerts are also effective data collected in the analysis processes by using the ecological environment improvement devices. The index data elated to the ecological improvement are collected, and the relevant feedback is given. The data obtained are used for the analysis on the performance of improvement in the ecological environment. The operational status of ecological environment improvements is analyzed to diagnose the causes of failures, which can also be used to monitor the causes of the relevant failures [27]. As shown in Figure 1, the environmental tax cost paid by enterprises based on clean technology is higher than the research and development cost. The technological innovation of enterprises based on clean technology has brought about the progress of clean technology and the improvement in the quality of clean technology products. However, the proportion of industries based on clean technology to the whole industry (as shown in the industrial structure variable in Figure 4 below) still presents a downward trend, and the features of economic structure optimization are not evident.

In the aspect of pollution emissions and pollution intensity, as the economic growth rate is decreased and the industrial structure has changed, the energy consumption of enterprises, especially those enterprises with substantial pollution emissions, has been reduced, and the total pollution emissions are also decreased accordingly. However, since the effect of environmental taxes on economic growth is more significant than its effect on pollution emissions, the pollution emission intensity still presents a slight upward trend in the end.

Based on different objectives, comparative studies of the effectiveness of producer price subsidies, consumer price subsidies, technology development subsidies, environmental tax policies, and other environmental control policies can also be implemented. Subsequently, the policies that have a more significant effect on improving social welfare are determined. Through research, the priority of different environmental control policies based on five objectives, that is, social welfare, economic growth, economic structure, environmental quality, and environmental technology, is obtained in this paper (as shown in Table 4).

In the aspect of economic growth and economic structure, price subsidies to producers have a relatively good effect, which is assessed from the production side where the manufacturing industry is regarded as the main body of the real economy in its development. Green growth is created based on the development needs of the real economy, and better quality green growth services can be provided to the manufacturing industry through the network platform and the green technology, so as to improve the market structure in the green growth. In the aspect of environmental quality and environmental technology, the subsidies for technology development should have the highest priority. As research and development investment is the main driver of technological progress, especially the enhancement of the green technology, the technological efficiency and technology level can truly be improved only by increasing the investment in research and development and carrying out the rational allocation of research and development resources. The advancement in green technology is in turn the main pathway to achieve cleaner production, lower pollutant emissions, and thus eliminating the relevant environmental problem. Hence, the direct role of subsidies for research and development in the technological advancement and its transmission effect in improving the environmental quality is very significant. The fundamental objective of environmental management is to achieve improvement in environmental quality while improving social welfare, that is, to achieve ecological and social benefits and to gain double dividends.

## 5. Conclusion

As China's economy enters a new normal, the downward pressure on economic growth has increased, and some local governments and enterprises are not committed enough to carry out environmental management properly. In this context, it is of tremendous theoretical and practical significance to study the environmental technologies and the stringency of environmental policies and their relationship with green growth in China. The development analysis on green growth has been extensively applied in the research on green growth development. For the purpose of further increasing the accuracy of the development analysis on the effect of environmental technology for green growth, a method for development analysis of environmental technology boosting the implementation of green growth is put forward in this paper. Based on this method, economic data and information on the objectives of environmental technology processes are collected, and the diversity of environmental technology processes present is taken into full account. The evolution of upgraded environmental technologies is analyzed in real time, and the evaluation algorithm is combined to carry out development analysis on the green growth based on environmental technologies. The method proposed in this paper can be used to analyze the green growth development in environmental technology process accurately and quickly. The result indicates that the environmental technology and the stringency of environmental policies have an indirect effect on the green growth in China through two pathways, that is, the technological innovation and the factor structure and FDI. This has demonstrated that the proposed method is relatively superior to the other analysis methods and can be used as a powerful tool for the subsequent analysis of environmental technologies.

## Figures and Tables

**Figure 1:** Pathway by which environmental technology and stringency of environmental policy affect the economic growth.

**Figure 2:** General framework of the green growth model in China.

**Figure 3:** Green growth across the country and in the three major regions (east, west, and central).

**Figure 4:** Policy effects of increasing the intensity of environmental taxes.

**Table 1:** Descriptive statistical analysis of various variables.

Symbols of variables	Minimum value	Maximum value	Mean value	Standard deviation	Definition of variables and source
GTFP	0.521	1.138	0.890	0.086	Calculation based on EBM-DDF
cer	0	28	3.622	4.559	Number of environmental regulations in each region^a^
lnmer	6.764	12.531	10.470	1.026	Total amount of sewage emission expenses in each region^a^
lnver	2.565	9.387	7.251	1.118	Number of environmental petitions and visits made by general public in each region^a^
TI	0.130	36.804	3.978	6.336	Number of patent applications granted per 10,000 people^b,c^
FS	0.010	0.228	0.057	0.029	Number of skilled labor force per unit of energy^d,e^
IS	0.494	3.658	0.901	0.448	Proportion of the output value in the tertiary industry divided by the output value in the secondary industry^f^
FDI	0.015	10.512	2.687	2.126	Proportion of foreign direct investment in GDP^c,f^

Data sources are annotated as the following: a: China Environment Yearbook; b: China Science and Technology Statistical Yearbook; c: China Statistical Yearbook; d: China Labor Statistical Yearbook; e: China Energy Statistical Yearbook; f: Statistical Yearbooks of various provinces.

**Table 2:** Direct effects of three environmental technologies and the stringency of environmental policies on green growth in China.

Variable	(I)cer	(II)mer	(III)ver	(IV)cer	(V)mer	(VI)ver
ER	0.001 (0.13)	0.031^*∗∗∗*^(3.10)	−0.010^∗^ (−1.75)	0.001 (0.08)	0.175^*∗∗*^ (2.19)	−0.137^*∗∗*^ (−3.37)
ER2				−0.0002 (−0.04)	−0.007^∗^ (−1.82)	0.009^*∗∗∗*^ (3.17)
Lnti	0.041^*∗∗∗*^ (3.66)	0.032^*∗∗∗*^ (3.17)	0.041^*∗∗∗*^ (4.07)	0.041^*∗∗∗*^ (3.59)	0.033^*∗∗∗*^ (3.19)	0.044^*∗∗∗*^ (4.47)
Lnfs	0.077^*∗∗*^ (2.37)	0.075^*∗∗∗*^ (2.72)	0.071^*∗∗*^ (2.49)	0.077^*∗∗*^ (2.36)	0.072^*∗∗∗*^ (2.63)	0.062^*∗∗*^ (2.22)
Lnis	0.052 (1.54)	0.063 (1.52)	0.074 (1.47)	0.052 (1.53)	0.058 (1.56)	0.087 (1.26)
Lnfdi	0.251^*∗∗*^ (2.29)	0.021^*∗∗*^ (2.21)	0.023^*∗∗*^ (2.44)	0.025^*∗∗*^ (2.27)	0.026^*∗∗*^ (2.61)	0.024^*∗∗*^ (2.52)
_cons	−0.315^*∗∗∗*^ (−2.89)	−0.635^*∗∗∗*^ (−4.25)	−0.225^*∗∗*^ (−2.32)	−0.318^*∗∗∗*^ (−2.88)	−1.315^*∗∗∗*^ (−3.27)	0.208 (1.25)
Hausman test *p* value	0.001	0.001	0.001	0.001	0.001	0.001
R-sq	0.813	0.717	0.772	0.813	0.725	0.768
F statistic quantity	32.13	42.64	40.15	26.67	36.34	36.06
Selection of the model	Fixed effects	Fixed effects	Fixed effects	Fixed effects	Fixed effects	Fixed effects
Sample size	360	360	360	360	360	360

The data in the parentheses are *t* statistic quantities, ^*∗*^, ^*∗*^, and ^*∗∗∗*^ indicate that it is significant at the levels of 10%, 5%, and 1%, respectively.

**Table 3:** Indirect effects of three environmental technologies and the stringency of environmental policies on green growth in China.

Variable	(I)cer	(Il)mer	(I)ver
LnER*∗*Lnti	0.019	0.002^*∗∗∗*^	0.006^*∗∗∗*^
	(1.24)	(2.49)	(4.87)

LnER*∗*Lnfs	0.015^*∗*^	0.010^*∗∗∗*^	0.003^*∗∗∗*^
	(1.80)	(4.50)	(1.98)

LnER*∗*Lnfdi	0.017^*∗∗*^	0.002^*∗∗*^	0.004^*∗∗∗*^
	(2.59)	(2.09)	(3.59)

_cons	−0.119^*∗∗∗*^	−0.392^*∗∗∗*^	−0.105^*∗∗*^
	(−11.9)	(−5.27)	(−2.57)

Hausman test *p* value	0.001	0.001	0.001
R-sq	0.693	0.751	0.767
F statistic quantity	14.35	64.24	61.10
Selection of the model	Fixed effects	Fixed effects	Fixed effects
Sample size	360	360	360

The data in the parentheses are *t* statistic quantities, ^*∗*^, ^*∗*^, and ^*∗∗∗*^ indicate that it is significant at the levels of 10%, 5%, and 1%, respectively.

**Table 4:** Comparative analysis of the effects of various policies for environmental regulation.

Objective	*Ranking of the effects of various policies for environmental regulation (effects arranged in a descending order)*			
	Best	Relatively good	General	Relatively weak
Economic growth	Subsidy to producers	Subsidy for research and development	Environmental tax	Subsidy to consumers
Economic structure	Subsidy to producers	Subsidy to consumers	Subsidy for research and development	Environmental tax
Social welfare	Subsidy to producers	Subsidy to consumers	Subsidy for research and development	Environmental tax
Environmental quality	Subsidy for research and development	Subsidy to consumers	Environmental tax	Subsidy to producers
Environmental technology	Subsidy for research and development	Subsidy to producers	Subsidy to consumers	Environmental tax

## Data Availability

The data used to support the findings of this study are available from the corresponding author upon request.
